# Effect of facet-joint degeneration on the in vivo motion of the lower lumbar spine

**DOI:** 10.1186/s13018-020-01826-z

**Published:** 2020-08-20

**Authors:** Jun Yin, Zhang Liu, Chao Li, Shiwei Luo, Qi Lai, Shaobai Wang, Bin Zhang, Zongmiao Wan

**Affiliations:** 1 Department of Orthopedics, The First Affiliated Hospital of Nanchang University, 17 Yongwai Street, Nanchang, Jiangxi 330006 PR China; 2 Science and Technology Office, The First Affiliated Hospital of Nanchang University, Nanchang, Jiangxi PR China; 3 Key Laboratory of Exercise and Health Sciences of Ministry of Education, School of Kinesiology, Shanghai University of Sport, Shanghai, China

**Keywords:** Facet-joint degeneration, Lumbar spine, In vivo motion, Vertebral kinematics, Spine biomechanics

## Abstract

**Objective:**

This research studied the in vivo motion characteristics of the L3–S1 lumbar spine with facet-joint degeneration during functional activities.

**Methods:**

Thirteen male and 21 female patients with facet-joint degeneration at the L3–S1 spinal region were included in the study. The L3–S1 lumbar segments of all the patients were divided into 3 groups according to the degree of facet-joints degeneration (mild, moderate, or severe). The ranges of motion (ROM) of the vertebrae were analyzed using a combination of computed tomography and dual fluoroscopic imaging techniques. During functional postures, the ROMs were compared between the 3 groups at each spinal level (L3–L4, L4–L5, and L5–S1).

**Results:**

At L3–L4 level, the primary rotations between the mild and moderate groups during left-right twisting activity were significantly different. At L4–L5 level, the primary rotation of the moderate group was significantly higher than the other groups during flexion-extension. During left-right bending activities, a significant difference was observed only between the moderate and severe groups. At L5–S1 level, the rotation of the moderate group was significantly higher than the mild group during left-right bending activity.

**Conclusions:**

Degeneration of the facet joint alters the ROMs of the lumbar spine. As the degree of facet-joint degeneration increased, the ROMs of the lumbar vertebra that had initially increased declined. However, when there was severe facet-joint degeneration, the ROMs of the lumbar spine declined to levels comparative to the moderate group. The relationship between the stability of the lumbar vertebra and the degree of facet-joint degeneration requires further study.

## Introduction

Lumbar facet joints are located in the posterior region of the vertebral column and are the only true synovial joints between adjacent spinal levels [1]. As part of the three-joint complex of the lumbar spine, the facet joint plays an important role in maintaining the stability and movement of the lower spine. In vitro studies have shown that these facet joints carry 6–30% of axial compressive loads during different activities [2]. This loading may also accelerate the degeneration of the lumbar facet joints. Facet-joint degeneration is prevalent among people over 60 years of age, and its severity is positively correlated with age [3]. In addition, facet-joint angles that have a greater sagittal orientation are closely associated with the risk of degeneration [4, 5]. Research has suggested that lumbar facet-joint degeneration occurs most commonly at the L4–L5 and L5–S1 levels [6].

Currently, the 4-grade criteria of Weishaupt et al. [7] is frequently adopted to evaluate facet-joint degeneration, and typical imaging has shown that narrow joint spaces are caused by thin cartilage, osteophytes, subchondral cysts, articular process hypertrophy, and subchondral bone sclerosis. The imaging classification of facet-joint degeneration plays an important role in clinical guidance as well. Traditional spinal-fusion surgery increases the risk of degeneration in adjacent segments, although spinal non-fusion surgeries such as intervertebral disc replacement and motion preservation device procedures may reduce the effects on adjacent spinal segments. However, the degree of lower back pain is related to the degree of facet degeneration in some patients, and simple disc replacement or interspinous process distractors may not completely relieve symptoms. Therefore, the classification of facet-joint degeneration is important for surgical decision-making.

Research had shown that facet-joint degeneration affects lumbar segment motion in vivo [8]. This research is, however, insufficient. Many studies on lumbar facet joints are aimed at individuals who have developed degenerative spinal diseases. Moreover, the degree of facet-joint degeneration has not been grouped. Therefore, the effect of facet joints with different degrees of degeneration on spinal movements remains unclear as the degree of degeneration of the facet joints varies depending on the segments involved and inconsistent force distributions.

To better understand the effect of different degrees of facet-joint degeneration on lumbar spine activity from a biomechanical perspective, we designed the current study based on computed tomography (CT) images by grouping the degree of facet-joint degeneration and comparing the ranges of motions (ROMs) of 7 functional activities on spinal levels L3 to S1. We hypothesized that the ROMs increase when facet-joint degeneration occurs. Our aim was to determine the effect of degree of facet joint degeneration on lumbar kinematics in vivo.

## Methods

Thirty-four patients (21 females and 13 males) hospitalized for degenerative spinal diseases (DSDs) were included in the study. All patients underwent lumbar spine CT and MRI examinations when admitted to the hospital. The age of the patients ranged from 33 to 73 years (Table 1). Approval of the experimental design was obtained by the appropriate Institutional Review Board prior to the initiation of the study. A written consent was obtained from each subject before the study.

**Table 1:** Demographics for the three groups of the facet joint degenerations at low lumbar spine

*BMI* body mass index

*One hundred two segments of 34 DDD patients were divided into three groups at L3–L4, L4–L5, and L5–S1 levels according to the facet degeneration Weishaupt’s grading

Exclusion criteria included the presence of other spinal diseases including lumbar spinal infection, fracture of the lumbar vertebrae, lumbar scoliosis with a Cobb angle larger than 10°, isthmic spondylolisthesis, and previous spinal surgery. The presence of back pain which affects lumbar movements taking about 15 min was used as indications for exclusion from the study. All CTs and MRIs were read by two senior spinal surgeons with > 15 years’ experience who were blinded to clinical patient information and the research hypothesis. The investigators independently read the CTs and MRIs in the same random order on a clinical Picture Archiving and Communication System (PACS) unit. When disagreements arose, another experienced radiologist (with over > 20 years’ experience) was consulted to provide consensus.

Facet-joint degeneration grading scores, facet sagittal angles, and disc degeneration degree were obtained from CT and MRI images. A number of studies have found a higher accuracy when evaluating facet joint degeneration with a CT image [9, 10]. In addition, Fujiwara et al. [11] showed that an MRI may underestimate the severity of osteoarthritis compared to CT images. Therefore, the degree of degeneration in the L3–S1 facet joints and discs were graded according to Weishaupt scales [7] and the Pfirmann classification [12], respectively. The degree of bilateral facet-joint degeneration was scored for each L3–S1 segment, and scores from 0 to 3 were matched to the grades of the same number. The scores from the left and right sides of the facet joints were summed and defined the 3 degeneration groups. Mild degeneration was scored from 1 to 2 points, moderate degeneration from 3 to 4 points, and severe degeneration from 5 to 6 points. The left and right facet-joint degeneration scores were usually either equal or differed by 1 point at each segment. However, there were 2 segments where one side had a score of 1and the other had a score of 3. In total, 102 segments from 34 DSD patients were divided into three groups at the L3–L4, L4–L5, and L5–S1 levels (Table 1).

### CT-based, three-dimensional (3D) geometric model of the vertebrae

To construct 3D lumbar-spine models of L3–S1, CT images (Fig. 1a) with a thickness of 0.75 mm, without a gap, and with a resolution of 512 × 512 pixels were imported into the modeling software program Mimics version 17.0 (Materialise, Leuven, Belgium) using an established, validated protocol [13].

**Fig. 1:** **a** A CT image of a human lumbar spine in the sagittal plane with segmentation lines present. **b** A 3-dimensional vertebral model from L3 to S1 constructed using CT images

### Dual fluoroscopic imaging and the establishment of virtual locations of vertebral positions

Following the completion of the 3D modeling (Fig. 1b), a dual fluoroscopic imaging system [14–16] was used to image the lumbar spines at different postures: upright standing position, maximum trunk flexion-extension, maximum left-right bending, and maximum left-right twisting (Fig. 2a). For subjects who experienced symptoms of lower back pain during functional activity, oral painkillers (Celebrex 200 mg) were administered to enable them to complete the 15-min exercises. Two fluoroscopes (Ziehm 8000; Ziehm imaging, Nuremberg, Germany) were positioned with their image intensifiers perpendicular to each other to obtain orthogonal images of the L3–S1 segments at different postures. The subjects remained still for several seconds during each target posture while the two fluoroscopes took images. To successfully image subjects while performing different postures, a distance of approximately 1 m was kept between the X-ray source and the receiver. To maximize the motion of the lower lumbar spine and maintain the spinal segments within the field of view of the two fluoroscopes, subjects were requested to minimize their hip movements.

**Fig. 2:** **a** Patients performing 7 functional activities of the trunk using a dual fluoroscopic imaging system. **b** Using the modeling software Rhinoceros 5.0, the in vivo vertebral activities were reconstructed

The in vivo motions of the lumbar spine at different functional positions were reproduced with the Rhinoceros version 5.0 modeling software (Robert McNeel & Associates, Seattle, WA, USA) (Fig. 2b) using the 3D vertebral models and orthogonal fluoroscopic images and an established protocol. Briefly, the CT image-based 3D models of the L3–S1 were independently translated and rotated in 6 degrees of freedom (6DOF) with increments of 0.01 mm and 0.01° until their outlines matched the osseous contours positioned on the 2 fluoroscopic images [13, 16].

### Relative motion measurements of the vertebrae

Right-handed Cartesian coordinate systems were used to quantify the 6DOF motions for the L3–S1 segments. In an upright position, the volumetric center of the vertebral body was chosen as the origin of the coordinate systems for each segment level. The x-axis was in the frontal plane and pointed in the left direction. The y-axis was in the sagittal plane and pointed in the posterior direction. The z-axis was vertical to the x–y plane and pointed proximally (Fig. 3a). Following reproduction of the in vivo vertebral positions, the motions of the lumbar vertebrae were measured from the coordinate system of the proximal vertebrae with respect to the distal vertebrae at the 3 vertebral levels: L3–L4, L4–L5, and L5–S1 (Fig. 3b). Three translations were defined as the motions of the proximal vertebral coordinate system origin in the distal coordinate system: anterior-posterior, left-right, and distal-proximal. The 3 rotations defined as the orientations of the proximal vertebral coordinate system in the distal vertebral coordinate system using Euler angles (in x–y–z sequence) were flexion-extension, left-right bending, and left-right twisting. The ROMs of L3–S1 were then determined from the ending ROM of flexion-extension, left-right bending, left-right twisting positions, and included both the primary translations and rotations, as well as the coupled translations and rotations in all 6 DOFs.

**Fig. 3:** **a** Local coordinate systems at the volumetric center of the vertebral body used to measure the relative motion of adjacent vertebra from L3–S1. **b** An example of vertebral motion measurements during flexion-extension activity

### Statistical analyses

Continuous variables were measured as means ± SDs, and a repeated measures ANOVA was used to compare the dynamic ROMs of the 3 facet-joint groups for all segment levels. When a statistically significant difference was detected, a post hoc Newman–Keuls test was performed. Statistical significance was set at *p* < 0.05. All statistical analyses were performed using the SPSS 24.0 statistical software (SPSS Inc., Chicago, IL, USA).

## Results

There were 102 vertebral segments from 34 patients with lumbar-spine degeneration disease that were divided into mild, moderate, and severe groups based on their facet-degeneration scores. There was no difference in the degeneration scores of the left and right facet joint in 67 segments, 33 segments of left and right facet-joint degeneration scores differ by 1 point, and 2 segments differ by 2 points. An analysis of study participant characteristics showed that patient BMI levels were not significantly different within or between the facet-joint groups and vertebral levels. However, there was a significant difference in patient ages between the mild, moderate, and severe facet-joint groups at all 3 segment levels, with the degree of degeneration increasing with patients age (*p* < 0.05). There was no significant difference in gender between the 3 groups at the different segment levels (Table 1).

No significant differences were found between the joint-facet degeneration grading scores and the 3 vertebral levels (*p* = 0.151). The sagittal angles of the facet joints increased with facet-joint degeneration at the L3–L4 level but were not significantly different. However, degeneration of the lumbar discs was correlated with facet-joint degeneration at the L3–L4 and L5–S1 levels. The L3–L4 disc-degeneration scores in the mild group was significantly lower than either the moderate (*p* < 0.01) or severe group (*p* = 0.014). There was also a significant difference between the mild and moderate groups at the L5–S1 level (*p* = 0.017) (Table 1).

### ROMs at the L3–L4 level

During flexion-extension activity, the primary rotations of the moderate facet-joint degeneration group showed a greater ROM compared to the mild and severe groups, but this difference was not statistically significant (Table 2; Fig. 4a). The coupled translation in the anterior-posterior directions in the moderate group was greater in comparison to the mild and severe group, but a significant difference was observed only between the mild and moderate groups (*p* = 0.044). The coupled motions in other directions were not significantly different (Table 2).

**Table 2:** Intervertebral 6DOF ROMs of L3–S1 with different facet-joint degeneration during functional activities

*L-R* left–right, *A-P* anterior–posterior, *P-D* proximal–distal translations, *F-E* flexion-extension bending, *Bend* left–right bending, *Twist* left–right twisting

**Fig. 4:** The range of primary rotations for different facet-joint degeneration categories at the L3–S1 levels during flexion-extension, left-right bending, and left-right twisting activities: **a** L3–L4; **b** L4–L5; **c** L5–S1. Asterisk and double asterisks represent statistical significance between group comparisons (*p* < 0.05, *p* < 0.01)

The primary ROMs of the mild, moderate, and severe groups during left-right bending activity were not significantly different nor were significant differences observed in the coupled motions (Fig. 4a).

During left-right twisting activity, the primary ROM of moderate group was larger than that of mild and severe group (Fig. 4a). However, a significant difference was found only between the mild and moderate groups (*p* = 0.040). There were no significant differences between the 3 groups for coupled translations and rotations.

### ROMs at the L4–L5 level

During flexion-extension activity, the primary rotations of the mild and severe groups were not significantly different (*p* = 0.630) (Fig. 4b), but both of these groups had lower ranges than the moderate group (*p* < 0.05). The coupled translation in the anterior-posterior direction of moderate group (2.6 ± 1.3 mm) was higher than the mild (1.5 ± 1.0 mm, *p* = 0.037) and severe groups (2.1 ± 1.0 mm, *p* > 0.05). The coupled translations in the left-right and proximal-distal directions were not significantly different nor were the coupled rotations in left-right bending and twisting axes.

During left-right bending activity, the primary rotations between the moderate (5.6 ± 2.2°) and severe groups (3.3 ± 1.5°) were statistically different (*p* = 0.008) (Fig. 4b). However, no significant differences were found between the coupled translations and rotations.

For left-right twisting activity, the primary rotations were not statistically different between the groups (*p* < 0.05) (see Table 2 and Fig. 4b). There were no significant differences observed for coupled motions.

### ROMs at the L5–S1 level

During flexion-extension activity, there was no significant difference in primary rotations (Fig. 4c) between the mild, moderate, and severe groups. However, coupled translations in the anterior-posterior direction were different between the 3 groups. The translation of the moderate group (3.4 ± 1.6 mm) was significantly greater than the mild (1.8 ± 1.2 mm) or severe (1.8 ± 1.3 mm) groups (*p* = 0.025 and *p* = 0.017, respectively). No significant differences were observed in the other coupled motions between the 3 groups.

During left-right bending activity, the primary rotations of the mild (2.8 ± 1.0°) and severe (4.6 ± 2.0°) groups were smaller than that of moderate group (3.0 ± 2.2) (Table 2). However, a significant difference was found only between the mild and moderate groups (*p* = 0.029) (Fig. 4c). The coupled translations and rotations were not significantly different.

For left-right twisting activities, no significant differences in primary rotations were found between the 3 groups, nor were there significant differences in coupled translations or rotations (Fig. 4c).

## Discussion

Previous studies of lumbar-spine kinematics have primarily focused on in vitro investigations. While in vivo studies have been undertaken [15, 17–19], few have taken into account weight-bearing conditions, motion patterns, or the degeneration level of the facet joints. The kinematic trends uncovered in this study were only partially consistent with previous studies due to different methods and research conditions. In Li et al.’s 2009 study [15], the authors investigated the ROMs of asymptomatic subjects at the L2–L3, L3–L4, and L4–L5 levels. While the ROMs at the L3–L4 and L4–L5 segments during flexion-extension activity in our experiment were similar to those reported by Li et al. for mild and severe groups, the ROMs of the moderate group were greater in our study. This difference may be due to the subjects in Li’s study performing 45° flexion and maximal extension as opposed to both maximal flexion and extension. In Li et al.’s study, coupled translations in proximal-distal direction were significantly lower at the L2–L3 as opposed to the L3–4 or L4–5 segments. This is in contrast to our data, where no differences in the translations were found between the levels. This may be due to the fact that our subjects retained some degree of facet-joint and disc degeneration that affected the ROM in the proximal-distal direction.

Few in vivo studies have reported the dynamic motion of the vertebrae during left-right bending activity. We found that the ROMs in our 3 groups at the L3–L4 level were greater than those found by Li et al. [15]. However, in the L4–L5 segment, the means of the mild and severe groups in our study were smaller. Their data also suggested that the rotation of the L4–L5 segment during this activity was significantly greater than for L2–3. However, the target segments of their study and ours are not exactly the same, and therefore, our results suggest that at the L3–4 level, vertebral mobility may have been increased due to facet-joint degeneration.

Our results also indicated that the ROMs between mild and moderate degeneration groups at the L3–L4 level were significantly different during left-right twisting activities. In the Li et al. study [15], the average twisting ranges for both the L3–L4 and L4–L5 levels were smaller in comparison to our results. In Passias et al.’s study [20], motions were observed in subjects with discogenic lower back pain using a combined imaging technique during flexion-extension, left-to-right bending, and left-to-right twisting movements. The ROMs found in their study were also smaller than our results, except at the L3–L4 level. These studies, along with our current results, indicate that facet-joint degeneration is related to the degeneration of the disc, and both have an effect on the left-right twisting movement of the vertebral body.

Shin et al. [21] investigated the in vivo characteristic motion patterns of the lumbar spine during dynamic axial rotation of the body. They found greater ranges of left-right twisting than we did. They also demonstrated that dynamic lumbar axial rotation coupled with lateral bending was segment dependent and created a coordinated dynamic coupling to maintain the global dynamic balance of the body. One possible reason for this difference may be because their subjects were asymptomatic. Other reasons may include differences in the participant age range and the male to female ratio. In particular, their subjects held weights to simulate daily functional activities during axial rotation. These additional loads may also be an important factor in explaining the differences in results.

Large discrepancies in vertebral rotation data may be due to different loading conditions and experimental designs [15]. In a study by Pearcy and Tibrewal [22], coupled translations in the anterior-posterior direction were found to be smaller than the average of the 3 groups in our study at the L3–S1 level and much smaller than the moderate group for the L3–S1 segments. Furthermore, we found that the translations between the mild and moderate degeneration groups were significantly different in the anterior-posterior direction during flexion-extension activity, and this phenomenon was found in all 3 segments. These horizontal and vertical comparisons indicate that weight-bearing and facet degeneration affect the coupled motions.

We also found differences in the vertebral kinematics caused by facet-joint degeneration, and an increasing trend in the average age of participants from the mild to severe degeneration groups. These findings are consistent with previous studies [1, 23]. Facet-joint degeneration is a progressive condition, which usually begins with changes in the articular cartilage and eventually leads to failure of the entire joint and an imbalance between the breakdown and repair of joint tissue. Researchers have suggested that the lumbar degenerative process can be categorized into three stages: temporary dysfunction, unstable, and restabilized [24]. This may explain the differences in the ROMs between the groups in our study. In patients with moderate facet-joint degeneration, the spine is in an unstable state, and when compared with mild degeneration, lumbar instability has reached a relatively high level. With further degeneration of the joint, its mobility will be strongly affected by the presence of osteophytes, which, in turn, will affect the activity of the lumbar spine. Our results suggest that this trend was present in all segments but was only significantly different in individual segments and positions.

Intervertebral discs and facets are closely related, and our data indicate that the degree of disc degeneration was significantly different between some of the groups at the L3–L4 and L5–S1 levels. While a strong relationship can be observed between discs and facet degeneration, it is difficult to assess a causal relationship, as many studies investigating this relationship have used cross-sectional designs. Some research has shown that facet degeneration typically follows disc degeneration [11]. Fujiwara et al. concluded that disc degeneration was closely associated with aging rather than facet-joint osteoarthritis [11]. Others have found facet-joint osteoarthritis in the absence of disc degeneration [25]. Although our results indicated a relationship between disc and facet-joint degeneration, a causal relationship could not be drawn, and the relationship remains controversial.

The transverse orientation of the lumbar facet joint is small, which enables a greater range of motion during flexion-extension activity. Our results indicate that the average transverse facet angle of each level (L3–S1) increases from the cephalad to caudad direction, which is consistent with previous findings [16].

This study has some limitations. First, the sample size was relatively small. This may explain the high variability between the groups. Second, we only analyzed the lumbar spine from L3 to S1. This was to focus on the lumbar segment where facet-joint degeneration is typically observed in the clinical setting. However, in future studies, the complete lumbar spine should be included. Finally, we only studied the end-point positions of each target activity, which may not be representative of the dynamic motion of the lumbar vertebrae.

## Conclusion

This study investigated the kinematics of the lower lumbar spine with varying degrees of facet-joint and disc degeneration. We found that mild to moderate facet-joint degeneration increased spinal mobility. However, when the joint was severely degenerated, the narrow joint space and proliferation of osteophytes restricted spinal movement, suggesting restabilization of the vertebrae may have occurred. These findings may serve as a reference for dynamic motion in degenerative spinal joint diseases and as a guide for timing surgical interventions.

## Data Availability

All data generated or analyzed during this study are included in the manuscript.

## Abbreviations

ROM: Ranges of motion
CT: Computed tomography
MRI: Magnetic resonance image
DSD: Degenerative spinal disease
6DOF: 6 degrees of freedom
